The article "A feed‐forward regulatory network lncPCAT1/miR‐106a‐5p/E2F5 regulates the osteogenic differentiation of periodontal ligament stem cells" was retracted in 2023. Reasons: errors in the images; duplicated images; unreliable results or conclusions.

# A feed‐forward regulatory network lncPCAT1/miR‐106a‐5p/E2F5 regulates the osteogenic differentiation of periodontal ligament stem cells

**DOI:** 10.1002/jcp.28550

**Published:** 2019-04-17

**Authors:** Bo Jia, Xiaoling Qiu, Jun Chen, Xiang Sun, Xianghuai Zheng, Jianjiang Zhao, Qin Li, Zhiping Wang

**Affiliations:** ^1^ Department of Oral Surgery Stomatological Hospital, Southern Medical University Guangzhou China; ^2^ Department of Plastic Surgery Guangzhou School of Clinical Medicine, Southern Medical University (Guangzhou General Hospital of Guangzhou Military Region) Guangzhou China

**Keywords:** periodontal ligament stem cells, prostate cancer‐associated ncRNA transcript‐1, miR‐106a‐5p, osteogenic differentiation, feed‐forward

## Abstract

Periodontal ligament stem cells (PDLSCs) are characterized by multiple differentiation potential and potent self‐renewal ability, yet much remains to be elucidated that what determines these properties. Long noncoding RNAs (lncRNAs) have been suggested to involve in multiple biological process under physiological and pathological conditions, including osteogenic differentiation. In the present study, we performed comprehensive lncRNA profiling by lncRNA microarray analysis and identified prostate cancer‐associated ncRNA transcript‐1 (lncPCAT1) was gradually increased in PDLSCs during consecutive osteogenic induction, and it could further positively regulate the osteogenic differentiation both in vitro and in vivo, whereas lncPCAT1 inhibition led to suppressed osteogenic differentiation*.* Thereafter, we inferred a predicted interaction between lncPCAT1 and miR‐106a‐5p and then confirmed the direct binding sites of miR‐106a‐5p on lncPCAT1. Although miR‐106a‐5p upregulation led to decreased osteogenic differentiation, lncPCAT1 overexpression could reverse its suppression, indicating that lncPCAT1 act as a competing endogenous RNA for miR‐106a‐5p. Moreover, lncPCAT1 could sponge miR‐106a‐5p to upregulate miR‐106a‐5p‐targeted gene BMP2, which was a crucial gene involved in osteogenic differentiation. Interestingly, we found that E2F5, another target of miR‐106a‐5p, could bind to the promoter of lncPCAT1 and then form a feed‐forward regulatory network targeting BMP2. In conclusion, our study provided a novel lncRNA‐miRNA feed‐forward regulatory network and a promising target to modulate the osteogenic differentiation of PDLSCs.

**Abbreviations**
ALP (ALPL): alkaline phosphatase
ARS: Alizarin red S
BMPs: bone morphogenetic proteins
ceRNA: competing endogenous RNA
HA‐TCP: hydroxyapatite‐tricalcium phosphate
HBMSCs: human bone‐marrow mesenchymal stem cells
HUMSCs: human umbilical cord‐derived mesenchymal stem cells.
lncRNAs: long‐noncoding RNAs
miRNAs: microRNAs
ncRNAs: noncoding RNAs
PCAT1: prostate cancer‐associated ncRNA transcript‐1
PDLSCs: periodontal ligament stem cells
RISC: RNA‐induced silencing complex

The article "A feed‐forward regulatory network lncPCAT1/miR‐106a‐5p/E2F5 regulates the osteogenic differentiation of periodontal ligament stem cells" was retracted in 2023. Reasons: errors in the images; duplicated images; unreliable results or conclusions.

## 1 INTRODUCTION

Chronic periodontitis is among the most common oral diseases, which causes loss of the supporting structure of the teeth including periodontal ligament, alveolar bone, and cementum (Anastasiadou, Jacob, & Slack, 2018; Reich & Hiller, 1993). Unlike other tissues, when it encounters inflammation, periodontal tissue cannot regenerate even after the alleviation of inflammation, partially due to the loss of differentiation capacity of periodontal ligament stem cells (PDLSCs) within the inflammatory microenvironment (Kamali, Korjan, Eftekhar, Malekzadeh, & Soufi, 2016; Xue et al., 2016). PDLSCs are derived from the periodontal ligament tissue, possess multiple differentiation potential and potent self‐renewal ability. These cells can further differentiate into bone, cartilage tissue and adipose tissue, and so forth (Seo et al., 2004). However, it has been reported that the capacity of PDLSCs was suppressed under inflammation and hypoxia (J. Zhang, Li, Si, Chen, & Meng, 2014), and could not be reversed even after remove of the stimulation on account of probable changes of several important signaling pathways (N. Liu et al., 2011). Some other reports revealed that growth factors, including Wnt family members (Cao et al., 2017; D. Liao, Li, Dong, & Sun, 2017; Wucheng et al., 2018) and bone morphogenetic proteins (BMPs; Hakki et al., 2014; Hyun, Lee, Kang, & Jang, 2017), transcription factors including β‐catenin (Chen et al., 2013; Li et al., 2016), and Runt‐related transcription factor 2 (RUNX2; Gao et al., 2013; He et al., 2018; Wei et al., 2017; Q. Zhou, Yang, Li, Liu, & Ge, 2016), as well as microRNA (W. Liu et al., 2013; Ng et al., 2015; Wei et al., 2017) could affect the osteogenic differentiation of PDLSCs. Further investigation into the regulation of PDLSCs during osteogenic differentiation might be promising to improve the osteogenic potential of PDLSCs and then regenerated the periodontal tissues.

Noncoding RNAs (ncRNAs) are a group of unique RNAs that have no protein‐coding properties but constitute almost 60% of the transcriptional output in human cells (Consortium, 2004; Djebali et al., 2012), and may involve in multiple cellular process, including cell proliferation, differentiation, and ontogenesis (Fedeli et al., 2016; Givel et al., 2018; Ismael, Altmeyer, & Stahl, 2016). There is a multitude of ncRNA species, including long noncoding RNAs (lncRNAs), which are longer than 200 nt in length, and microRNAs (miRNAs; Anastasiadou et al., 2018). Both these two types of ncRNAs have been reported to be involved in osteogenic differentiation under normal and aberrant conditions. For instance, lncRNAs such as TUG1, H19, and MEG3 could promote osteogenesis in several kinds of stem cells (He et al., 2018; J. Liao, Yu, et al., 2017; Zhuang et al., 2015), whereas inhibition of lncRNA MIR31HG in human adipose‐derived stem cells may promote osteogenic differentiation (Jin et al., 2016). Beyond analyzing their functions in isolation, a regulatory network composed of lncRNA and miRNA exhibits more significant role in regulation of cellular process (Anastasiadou et al., 2018). miRNAs naturally regulate the expression of messenger RNAs (mRNAs) by directly binding to their 3′‐untranslated regions (3′‐UTRs), while lncRNAs can then act as a sponge and regulate the abundance of miRNAs through segregating this process (Beermann, Piccoli, Viereck, & Thum, 2016; Lu & Zhao, 2017; Qu et al., 2016). It has been reported that lncRNA TUG1 could sponge miR‐204‐5p and then promote osteogenic differentiation through upregulating RUXN2 (C. Yu, Li, et al., 2018).

The article "A feed‐forward regulatory network lncPCAT1/miR‐106a‐5p/E2F5 regulates the osteogenic differentiation of periodontal ligament stem cells" was retracted in 2023. Reasons: errors in the images; duplicated images; unreliable results or conclusions.

The role of prostate cancer‐associated ncRNA transcript‐1 (lncPCAT1) has been thoroughly discussed in several kinds of cancers (Bi, Yu, Huang, & Tang, 2017; Shen et al., 2017; Shi et al., 2015). Recent study has verified its promoting effect in osteogenic differentiation of adipose‐derived stem cells via activating the TLR signalling pathway (L. Yu, Qu, et al., 2018), inspiring us to further explore its role and regulatory mechanisms in osteogenic differentiation of PDLSCs. In the present study, we have found that lncPCAT1 was involved in PDLSCs osteogenesis, and positively regulated the osteogenic differentiation of PDLSCs. During this process, lncPCAT1 sponged miR‐106a‐5p and formed a mutual regulatory network targeting BMP2 and E2F5. Interestingly, we found E2F5 in turn promoted the transcription of lncPCAT1, forming a feed‐forward loop. It is the first report, to our knowledge, that demonstrates the regulation of osteogenic differentiation of PDLSCs by lncPCAT1‐miR‐106a‐5p‐E2F5 feed‐forward loop regulatory network.

## 2 MATERIALS AND METHODS

### 2.1 Cell cultures

The periodontal ligament stem cells (PDLSCs), human bone‐marrow mesenchymal stem cells (HBMSCs), and human umbilical cord‐derived mesenchymal stem cells (HUMSCs) were purchased from Salila (Guangzhou, China). The cells were cultured in growth medium (GM) consisting of DMEM (Gibco, Grand Island, NY) supplemented with 10% fetal bovine serum (Gibco) at 37℃ in a humidified atmosphere of 5% CO_2_. For osteogenic induction, the PDLSCs were cultured with osteogenic medium (OM) consisting of growth medium, 100 mmol/L dexamethasone (Sigma‐Aldrich; Merck KGaA, Damstadt, Germany), 0.05 mmol/L ascorbate acid (Sigma‐Aldrich; Merck KGaA), and 10 mmol/L β‐glycerophosphate (Sigma‐Aldrich; Merck KGaA). The medium was changed every 2 days. For another differentiation of the PDLSC cells, chondrogenic differentiation medium (Cyagen, Guangzhou, China) or adipogenic differentiation medium (Cyagen) were applied.

The article "A feed‐forward regulatory network lncPCAT1/miR‐106a‐5p/E2F5 regulates the osteogenic differentiation of periodontal ligament stem cells" was retracted in 2023. Reasons: errors in the images; duplicated images; unreliable results or conclusions.

### 2.2 Microarray

Two samples (PDLSCs and osteogenic‐induced PDLSCs), each contained 1 × 10^6^ cells were prepared, and total RNA was isolated and purified with an RNeasy mini kit (Cat. #74106; Qiagen, Hilden, Germany). Each slide was hybridized with 1.65 μg Cy3‐labeled cRNA using a Gene Expression Hybridization Kit (Cat. #5188–5242; Agilent Technologies, Palo Alto, CA) in a hybridization oven (Cat. #G2545A;Agilent Technologies). The process of hybridization was last for 17 hr and washed in staining dishes (Cat. #121; Thermo Fisher Scientific, Waltham, MA) with a Gene Expression Wash Buffer Kit (Cat. #5188–5327; Agilent Technologies). Then the slides were scanned with an Agilent Microarray Scanner (Cat. #G2565CA; Agilent Technologies) followed by the default settings: dye channel, green; scan resolution, 3 μm; PMT, 100%; 20 bit. Feature Extraction software 10.7 (Agilent Technologies) was used for data extracting. A microarray analysis was performed by Shanghai Biotechnology Cooperation (Shanghai, China).

### 2.3 ALP activity assay

The transfected PDLSCs were cultured with osteogenic induction medium for 7 days in 24‐well plates at a density of around 1 × 10^5^ cells/well, then the ALP activity was measured by ALP activity kit according to the protocol (Nanjing Jiancheng, Nanjing, China).

### 2.4 Mineralization assay

The transfected PDLSCs were cultured with osteogenic induction medium for 7 days in 24‐well plates at a density of around 1 × 10^5^ cells/well, and the mineralization of the PDLSCs was observed via Alizarin red S (ARS) and alkaline phosphatase (ALP) staining according to the manufacture's protocols (ARS staining kit; Solarbio, Beijing, China; ALP staining kit; Nanjing Jiancheng, China).

### 2.5 Western blot analysis

Total protein was extracted from the cells by lysis with radioimmunoprecipitation assay buffer (DGCS Biotechnology, Beijing, China). The protein content of the lysate was then determined using the BCA kit (Beyotime, Shanghai, China) according to the manufacturer's protocol. Then, 20 μg of the cell lysate were separated by 10% sodium dodecyl sulfate polyacrylamide gel electrophoresis, and the separated proteins were transferred to a polyvinylidene fluoride membrane (Millipore, MA). The membranes were blocked with 5% BSA for 2 hr and then incubated with primary antibodies over night at 4°C. Primary antibodies are listed as follows: RUNX2 (1:1,000; Cell Signaling Technology, Danvers, MA), Osterix (OSX; 1:1,000; Abcam, Cambridge, UK), glyceraldehyde 3‐phosphate dehydrogenase (1:1,000; Cell Signaling Technology), E2F5 (1:2,000; Abcam), BMP2 (1:1,000; Cell Signaling Technology), Smad5 (1:1,000; Cell Signaling Technology), and p‐Smad5 (1:1,000; Cell Signaling Technology). The immune complexes were then immunoblotted with an HRP‐conjugated anti‐mouse or anti‐rabbit immunoglobulin‐G (IgG) antibody (1:2,000; CWBio, Beijing, China). Immunodetection was performed using the enhanced chemiluminescence reagents (Fdbio, Hangzhou, China). All experiments were repeated three times.

The article "A feed‐forward regulatory network lncPCAT1/miR‐106a‐5p/E2F5 regulates the osteogenic differentiation of periodontal ligament stem cells" was retracted in 2023. Reasons: errors in the images; duplicated images; unreliable results or conclusions.

### 2.6 RNA isolation and reverse transcription quantitative polymerase chain reaction (RT‐qPCR) analysis

Total RNA was extracted with TRIzol reagent(Invitrogen, Thermo Fisher Scientific) and converted into cDNA (Invitrogen, Thermo Fisher Scientific). The miR‐106a‐5p were reverse‐transcribed using a specific RT primer (RiboBio, Guangzhou, China) according to the manufacturer's protocol. β‐Actin was used as endogenous normalization control for messenger RNA (mRNAs) and lncRNAs. U6 was used as endogenous normalization control for miR‐106a‐5p. Primer pairs for all lncRNAs and miRNAs were designed by RiboBio. RT‐qPCR was performed using the SYBR Green PCR Kit (Toyobo, Osaka, Japan) and the Applied Biosystems 7500 Real‐Time PCR Detection System (Life Technologies Corporation, Carlsbad). The data were analyzed using the $2^{-{\Delta \Delta C}_{t}}$ relative expression method. All experiments were repeated three times. Primer sequences were listed in Supporting Information.

### 2.7 Oligonucleotide, plasmids, and cell transfection

Both the siRNAs, miRNA mimics, miRNA inhibitors were purchased from RiboBio. The plasmids were purchased from GeneChem (Shanghai, China). Oligonucleotide and plasmids transfection was conducted using Lipofectamine 2000 transfection reagent (Invitrogen; Thermo Fisher Scientific, Waltham, MA) following the manufacturer's protocol. After 48 hr of transfection, the cells were collected and used for further examinations.

### 2.8 Lentiviruses and cell transfection

All the plasmids and lentiviruses were designed and constructed by GeneChem. PDLSCs were cultured at a concentration of 2 × 10^5^ cells/well in six‐well plates. After the cells had grown to 30–40% confluence, they were transfected with lentiviruses in the presence of polybrene.

### 2.9 In vivo transplantation

The NOD/SCID mice around 4‐week old purchased from Provincial Animal Center (Guangdong, China) were randomly divided into four groups with five mice per group. For the transplantation, around 5 × 10^6^ cells were loaded onto 20 mg hydroxyapatite‐tricalcium phosphate scaffold (HA‐TCP; Sigma, St. Louis, MO) and subcutaneously implanted into the dorsal region of NOD/SCID mice. General anesthesia was performed by intraperitoneal injection of pentobarbital sodium (0.1 ml/100 g) for all surgical procedures. All animal procedures were approved by the Animal Care Committee of Southern Medical University. After 4 weeks, the mice were killed by cervical dislocation under general anesthesia. The xenografts were removed, fixed with 4% paraformaldehyde and decalcified in 10% ethylenediaminetetraacetic acid (pH 6.0) for 7 days. For histological analyses, the xenografts were then embedded in paraffin, sectioned and stained with hematoxylin and eosin (H&E; Beyotime Institute of Biotechnology, Shanghai, China), or Masson's Trichrome stain (Sigma‐Aldrich; Merck KGaA), according to the protocols of manufacturer.

The article "A feed‐forward regulatory network lncPCAT1/miR‐106a‐5p/E2F5 regulates the osteogenic differentiation of periodontal ligament stem cells" was retracted in 2023. Reasons: errors in the images; duplicated images; unreliable results or conclusions.

### 2.10 RNA immunoprecipitation

RIP assay was performed using an RNA Binding Protein Immunoprecipitation Kit (Millipore) according to the manufacturer's protocols with an anti‐Ago2 antibody (1:1,000; Abcam) or normal mouse IgG as a negative control. RT‐qPCR was then performed as described above. All experiments were repeated three times.

### 2.11 Luciferase reporter assay

The putative miR‐106a‐5p binding sites in lncPCAT1, E2F5, and BMP2, both wild‐type and mutant type, were synthesized and cloned downstream of the luciferase gene in pmirGLO luciferase vectors (Genechem). The plasmids, miRNA mimics (miR‐NC and miR‐106a‐5p), miRNA inhibitor (control anti‐miRNA, anti‐ miR‐106a‐5p) and Renilla luciferase plasmid (Genechem), used as a normalization control, were cotransfected into cells using Lipofectamine 2000 (Invitrogen). Firefly and Renilla luciferase activities were then measured consecutively by Dual Luciferase Assay 48 hr after transfection. All experiments were repeated three times.

### 2.12 Chromatin immunoprecipitation (ChIP) assay

ChIP was conducted using EZ‐ChIP Kit (Millipore) as previously reported (Fang et al., 2016). PDLSCs cell chromatin was immunoprecipitated using anti‐E2F5 (Abcam) antibody. Anti‐IgG (Millipore) antibody was used as a negative control. Fold enrichment was determined by RT‐qPCR and calculated as a percentage of anti‐IgG group (E2F5/IgG). Sequences of primers used for RT‐qPCR in this study were listed as follows: predicted binding site (BD): sense primer 5′‐TGAGTTGGGCTTTGCTTGTT‐3′, and antisense primer 5′‐TTTAGGGCACTAATGATTTCTTATC‐3′; negative control (NEG): sense primer 5′‐CTCTAGCTAACTGTGATCAGGCTGG‐3′, and antisense primer 5′‐CCAGCCTGATCACAGTTAGCTAGAG‐3′.

The article "A feed‐forward regulatory network lncPCAT1/miR‐106a‐5p/E2F5 regulates the osteogenic differentiation of periodontal ligament stem cells" was retracted in 2023. Reasons: errors in the images; duplicated images; unreliable results or conclusions.

### 2.13 Statistical analysis

All statistical analyses in this study were performed with SPSS 16.0 software (SPSS Inc., Armonk, NY). Data are presented as the mean ± *SD*. The significance of mean values between two groups were analyzed using two‐tailed unpaired Student's *t* test. Differences in multiple groups were determined by one‐way analysis of variance with subsequent Bonferroni correction. Pearson's product‐moment correlation coefficients were used to analyze the correlation of the two variables. *p* Value <0.05 was considered statistically significant.

## 3 RESULTS

### 3.1 The expression of lncPCAT1 was significantly altered during osteogenic induction and was correlated with osteogenic differentiation of PDLSCs

To induce osteogenic differentiation, the PDLSCs were treated with osteogenic differentiation medium. High‐throughput sequencing was applied to detect lncRNAs after osteogenic differentiation of PDLSCs. A heatmap describing the changes in lncRNAs was shown in Figure 1a. We confirmed the microarray results using RT‐qPCR and found NR_045262 (lncPCAT1) was the most significantly altered lncRNA between the non‐induced group and osteogenic‐induced group (Figure 1b). The expression of lncPCAT1 and three osteogenic genes, including RUNX2, OSX, and ALPL, were then determined in PDLSCs at 0, 3, 7, 14, and 21 days after osteogenic induction, and found to be gradually increasing during the induction. In comparison, the expression of these genes seemed unchanged under growth medium (Figure 1c). Subsequently, positive correlations between the levels of lncPCAT1 and other three genes were found (Figure 1d), indicating the potential involvement of lncPCAT1 during osteogenic induction.

**Figure 1:** The expression of lncPCAT1 was significantly altered during osteogenic induction and was correlated with osteogenic differentiation of PDLSCs. (a) Heatmap of differentially expressed lncRNAs (the top 20 in upregulated lncRNAs and the top 20 in downregulated lncRNAs) between GM‐ and OM‐treated PDLSCs for 14 days. (b) The top 10 in upregulated lncRNAs were confirmed by RT‐qPCR (*n* = 3). (c) The mRNA levels of lncPCAT1, RUNX2, OSX, and ALPL were determined in PDLSCs at 0, 3, 7, 14, and 21 days under OM and GM by RT‐qPCR (*n* = 3). (d) Correlation analysis was performed between lncPCAT1 level and RUNX2, OSX, and ALPL mRNA levels in PDLSCs at 0, 3, 7, 14, and 21 days after osteogenic induction. Data represent mean ± *SD*. *p <0.05, **p <0.01. ALPL: alkaline phosphatase; GM: growth medium; lncPCAT1: prostate cancer‐associated ncRNA transcript‐1; lncRNAs: long noncoding RNAs; mRNA: messenger RNA; OM: osteogenic medium; OSX: osterix; PDLSCs: periodontal ligament stem cells; RT‐qPCR: reverse transcription quantitative polymerase chain reaction [Color figure can be viewed at wileyonlinelibrary.com]

The article "A feed‐forward regulatory network lncPCAT1/miR‐106a‐5p/E2F5 regulates the osteogenic differentiation of periodontal ligament stem cells" was retracted in 2023. Reasons: errors in the images; duplicated images; unreliable results or conclusions.

### 3.2 lncPCAT1 promoted osteogenic differentiation of PDLSCs both in vitro and in vivo

To determine the role of lncPCAT1 on the osteogenic differentiation of PDLSCs, we constructed two different lentiviral plasmids for lncPCAT1 knockdown (shPCAT1‐1 and shPCAT1–2) and a lncPCAT1‐overexpressing lentiviral plasmid (lncPCAT1). The transfection effect was then confirmed by RT‐qPCR (Figure 2a). Since positive correlations between lncPCAT1 and osteogenic genes, we then detected the expression of RUNX2, OSX, and ALPL after 7 days osteogenic induction in transfected PDLSCs and found that lncPCAT1 overexpression significantly upregulated the mRNA levels of RUNX2, OSX, and ALPL in PDLSCs, whereas knockdown of lncPCAT1 significantly downregulated the expression of these genes (Figure 2b–d). The regulation of lncPCAT1 on RUNX2 and OSX was further confirmed at protein level (Figure 2e). To further investigate the effects of lncPCAT1 on osteogenic process, ALP activity assay, Alizarin red S (ARS) staining and alkaline phosphatase (ALP) staining were performed and revealed that lncPCAT1 overexpression increased ALP activity and mineralized bone matrix formation in PDLSCs. Conversely, they were significantly decreased upon lncPCAT1 knockdown (Figure 2f,g). We further evaluated the effect of lncPCAT1 on PDLSCs osteogenesis in vivo. The transfected PDLSCs loaded with HA‐TCP were subcutaneously implanted in the dorsal region of NOD/SCID mice. After 4 weeks, the implants were removed and the newly formed bone tissue was then stained with H&E stain and Masson's trichrome stain. Comparing to the negative control, lncPCAT1 overexpression led to increased osteoid formation. Contrarily, knockdown of lncPCAT1 resulted in decreased osteoid formation (Figure 2h). Interestingly, the lncPCAT1 level in PDLSCs was neither increased when differentiated into adipose cells nor induced into chondrocytes (Figure S1A). While the ARS or alkaline phosphatase (ALP) staining showed the same trend in both HBMSCs and HUMSCs, suggesting lncPCAT1 involved in promoting osteogenic differentiation specifically (Figure S1B,C). In conclusion, these results showed that lncPCAT1 could promote osteogenic differentiation of PDLSCs both in vitro and in vivo.

**Figure 2:** LncPCAT1 promoted osteogenic differentiation of PDLSCs both in vitro and in vivo. (a) Transfection effects of lncPCAT1 silence and overexpression in PDLSCs were determined by RT‐qPCR (*n* = 3). (b–d) The mRNA levels of RUNX2, OSX, and ALPL were determined in transfected PDLSCs at 7 days after osteogenic transduction by RT‐qPCR (*n* = 3). (e) The protein levels of RUNX2 and OSX were determined in transfected PDLSCs at 7 days after osteogenic transduction by Western blot analysis. (f,g) ALP activity assay, ARS staining and ALP staining were measured in lncPCAT1 overexpressed or silenced PDLSCs at 7 days after osteogenic transduction. (h) Transfected PDLSCs after 7 days osteogenic differentiation loaded on HA‐TCP were transplanted into the dorsal region of NOD/SCID mice, and the xenografts were removed and stained with H&E and Masson's Trichrome stain, respectively (*n* = 5 per group). All experiments were repeated three times. Data represent mean ± *SD*. *p  < 0.05, **p  < 0.01. ALPL: alkaline phosphatase; HA‐TCP: hydroxyapatite‐tricalcium phosphate; lncPCAT1: prostate cancer‐associated ncRNA transcript‐1; NC: negative control; OSX: osterix; PDLSCs: periodontal ligament stem cells; RT‐qPCR: reverse transcription quantitative polymerase chain reaction; RUNX2: Runt‐related transcription factor 2 [Color figure can be viewed at wileyonlinelibrary.com]

The article "A feed‐forward regulatory network lncPCAT1/miR‐106a‐5p/E2F5 regulates the osteogenic differentiation of periodontal ligament stem cells" was retracted in 2023. Reasons: errors in the images; duplicated images; unreliable results or conclusions.

### 3.3 LncPCAT1 acted as a sponge of miR‐106a‐5p

To determine whether lncPCAT1 acted as a miRNA sponge that competed with mRNA for binding to miRNAs, we used lncRNABase (www.lncrnadb.org) and NONCODE (www.noncode.org), and found two putative binding sites of miR‐106a‐5p to lncPCAT1 (Figure 3a). miR‐106a has been reported to be involved in the osteogenic differentiation of cell (Li et al., 2013). Based on this prediction, luciferase reporter constructs carrying lncPCAT1 reporter were generated. The results revealed that the lncPCAT1‐wt reporter and lncPCAT1‐mut1 reporter were strongly inhibited by miR‐106a‐5p, whereas lncPCAT1‐mut2 reporter was not affected by miR‐106a‐5p (Figure 3b,c), indicating that miR‐106a‐5p directly bond to lncPCAT1 at the predicted binding site 1. We also confirmed that lncPCAT1 was associated with the RNA‐induced silencing complex (RISC) by RNA‐binding protein immunoprecipitation assay, indicating the potential relationship between lncPCAT1 and miR‐106a‐5p (Figure 3d). Furthermore, we found a gradual decrease of miR‐106a‐5p in PDLSCs during osteogenic induction (Figure 3e), a negative correlation between the miR‐106a‐5p expression and lncPCAT1 expression during the osteogenic induction was confirmed (Figure 3f). In addition, miR‐106a‐5p level was decreased following lncPCAT1 overexpression and lncPCAT1 silence led to increased level of miR‐106a‐5p in PDLSCs (Figure 3g).

**Figure 3:** LncPCAT1 acted as a sponge of miR‐106a‐5p. (a) Schematic diagram of the miR‐106a‐5p putative binding sites and mutant site in lncPCAT1. (b, c) The target validation using luciferase reporters in PDLSC cells (*n* = 3). The relative luciferase activities of luciferase reporters containing WT or Mut transcripts were assayed in miR‐106a‐5p overexpressed or silenced PDLSCs. (d) Association of lncPCAT1 and miR‐106a‐5p with Ago2 pulldown assay (*n* = 3). Cellular lysates from PDLSC cells were used for RNA immunoprecipitation with Ago2 antibodies. the levels of lncPCAT1 and miR‐106a‐5p were detected using RT‐qPCR. (e) The level of miR‐106a‐5p was determined in PDLSCs at 0, 3, 7, 14 and 21 days under OM and GM by RT‐qPCR (*n* = 3). (f) Correlation analysis was performed between miR‐106a‐5p level and lncPCAT1 level at indicated time after osteogenic induction. (g) The level of miR‐106a‐5p in lncPCAT1 overexpressed or silenced PDLSCs was determined by RT‐qPCR (*n* = 3). Data represent mean ± *SD*. *p <0.05, **p  < 0.01, ***p < 0.001. lncPCAT1: prostate cancer‐associated ncRNA transcript‐1; miR: microRNA; mut: mutant; NC: negative control; PDLSCs: periodontal ligament stem cells; WT: wild‐type [Color figure can be viewed at wileyonlinelibrary.com]

The article "A feed‐forward regulatory network lncPCAT1/miR‐106a‐5p/E2F5 regulates the osteogenic differentiation of periodontal ligament stem cells" was retracted in 2023. Reasons: errors in the images; duplicated images; unreliable results or conclusions.

### 3.4 LncPCAT1 could negatively regulate miR‐106a‐5p during osteogenic induction

It was previously reported that miR‐106a involved in the osteogenic differentiation. Consistent with this finding, miR‐106a‐5p mimics decreased the RUNX2, OSX, and ALPL mRNA levels and miR‐106a‐5p inhibitor increased these levels (Figure 4a–d). As lncPCAT1 could act as a sponge of miR‐106a‐5p, we subsequently investigated how this interaction affects the osteogenic differentiation. Consistently, miR‐106a‐5p upregulation could reverse the effect of lncPCAT1 on RUNX2, OSX, and ALPL levels at 7 days after osteogenic induction (Figure 4e–h). Moreover, the cotransfected PDLSCs was measured using ALP activity assay, ARS staining and ALP staining after osteogenic induction, and the negative regulation between lncPCAT1 and miR‐106a‐5p was also observed (Figure 4i,j).

**Figure 4:** LncPCAT1 could negatively regulate miR‐106a‐5p during osteogenic induction. (a) The transfection effects of miR‐106a‐5p mimics and inhibitors were confirmed by RT‐qPCR (*n* = 3), respectively. (b–d) The mRNA level of RUNX2, OSX, and ALPL in miR‐106a‐5p transfected PDLSCs at 7 days after osteogenic transduction (*n* = 3). (e–h) lncPCAT1 overexpressed PDLSCs were transfected with miR‐106a‐5p mimics, and the expressions of RUNX, OSX, and ALPL at 7 days after osteogenic induction were determined by RT‐qPCR and Western blot analysis (*n* = 3). (i, j) Osteogenic differentiation was determined in transfected PDLSCs at 7 days after osteogenic transduction by ALP activity assay, ARS staining and ALP staining. Data represent mean ± *SD*. *p <0.05, **p <0.01. ALPL, ALP: alkaline phosphatase; lncPCAT1: prostate cancer‐associated ncRNA transcript‐1; miR: microRNA; mRNA: messenger RNA; NC: negative control; OSX: osterix; PDLSCs: periodontal ligament stem cells; RUNX2: Runt‐related transcription factor 2 [Color figure can be viewed at wileyonlinelibrary.com]

The article "A feed‐forward regulatory network lncPCAT1/miR‐106a‐5p/E2F5 regulates the osteogenic differentiation of periodontal ligament stem cells" was retracted in 2023. Reasons: errors in the images; duplicated images; unreliable results or conclusions.

### 3.5 BMP2 was a target of lncPCAT1/miR‐106a‐5p regulatory network during osteogenesis

Analysis of the downstream targets of miR‐106a‐5p using both TargetScan (http://www.targetscan.org) and microT‐CDS (http://diana.imis.athena‐innovation.gr) showed totally 137 common target genes (Figure 5a), including BMP2, which was previously reported to be involved in osteogenic differentiation (Manochantr et al., 2017). Consistent with this report, binding site of miR‐106a‐5p in BMP2 was confirmed using luciferase reporter assay (Figure 5b–d). Protein levels of BMP2 and phosphorylated Smad5, a downstream regulated target of BMP2 in the osteogenic differentiation of cells (Retting, Song, Yoon, & Lyons, 2009), was decreased in PDLSCs transfected with miR‐106a‐5p mimics, whereas they were increased by miR‐106a‐5p inhibitor (Figure 5e). In parallel, the mRNA expression of BMP2 showed the same tendency (Figure S2A). Likewise, the mRNA level of BMP2 gradually increased in PDLSCs during continuous osteogenic induction (Figure S2B), and negatively correlated with the level of miR‐106a‐5p (Figure S2C). The positive regulation of lncPCAT1 on BMP2 was also determined (Figure S2D,E). Overexpression of lncPCAT1 in PDLSCs cells led to the increased enrichment of Ago2 on lncPCAT1 but substantially decreased enrichment on BMP2 transcripts. In parallel, lncPCAT1 knockdown elicited a significant increase in the recruitment of Ago2 to BMP2 transcripts compared with control cells, suggesting that lncPCAT1 could compete with BMP2 transcripts for the Ago2‐based miRNA‐induced repression complex (Figure 5f,g). This effect was also verified by Western blot analysis and qRT‐PCR (Figure S2F,G). The impacts of BMP2 on osteogenic process were further determined. Inhibition of BMP2 dramatically decreased RUNX2 and phosphorylation of Smad5 expression after osteogenic induction (Figure 5l), meanwhile, osteoblast‐related gene was also decreased (Figures 5h and S2H). ALP activity assay along with ARS and ALP staining further confirmed the promotion of BMP2 on osteogenesis (Figure 5i,j). What's more, knockdown of BMP2 decreased the osteoid formation in vivo (Figure 5k).

**Figure 5:** BMP2 was a target of lncPCAT1/miR‐106a‐5p regulatory network during osteogenesis. (a) Target genes predicted by TargetScan and microT‐CDS were selected as potential target genes of miR‐106a‐5p. (B) Schematic diagram of the miR‐106a‐5p putative binding sites in wild‐type and mutant BMP2 3′‐UTR. (c, d) The binding sites of miR‐106a‐5p to wild‐type or mutant BMP2 3′‐UTR under transfection with miR‐106a‐5p mimics or inhibitors were determined with luciferase reporter assay (*n* = 3). (e) The protein levels of BMP2, p‐Smad5, and t‐Smad5 were determined in PDLSCs transfected with miR‐106a‐5p mimics or inhibitor by Western blot analysis. (f, g) RIP assay of the enrichment of Ago2 on lncPCAT1, BMP2 transcripts relative to IgG in PDLSC cells transfected with lncPCAT1 overexpression or silence lentivirus and their corresponding controls (*n* = 3). (h) The protein levels of BMP2, RUNX2, p‐Smad5, and t‐Smad5 in sh‐BMP2 transfected PDLSCs at 7 days after osteogenic induction were determined by Western blot analysis. (i, j) Osteogenic differentiation of PDLSCs transfected with sh‐BMP2 was determined by ALP activity, ARS, and ALP staining at 7 days after osteogenic induction. (k) H&E and Masson staining were performed in BMP2 silenced PDLSCs in vivo (*n* = 5 per group). Data represent mean ± *SD*. *p <0.05, **p <0.01. 3′‐UTR: 3′‐untranslated region; Ago2: argonaute 2; ALP: alkaline phosphatase; ARS: Alizarin red S; BMP2: bone morphogenetic protein 2; H&E: hematoxylin and eosin; lncPCAT1: prostate cancer‐associated ncRNA transcript‐1; miR: microRNA; NC: negative control; PDLSCs: periodontal ligament stem cells; RIP: RNA‐binding protein immunoprecipitation; RUNX2: Runt‐related transcription factor 2 [Color figure can be viewed at wileyonlinelibrary.com]

The article "A feed‐forward regulatory network lncPCAT1/miR‐106a‐5p/E2F5 regulates the osteogenic differentiation of periodontal ligament stem cells" was retracted in 2023. Reasons: errors in the images; duplicated images; unreliable results or conclusions.

### 3.6 E2F5 could also promote osteogenesis under the regulation of lncPCAT1/miR‐106a‐5p

Among the 137 miR‐106a‐5p directly‐targeted genes mentioned above, E2F5 was the only transcription factor predicted (Figure 6a). Interestingly, E2F5 was predicted to bind to the promoter region of lncPCAT1 using PROMO database (http://alggen.lsi.upc.es/cgi‐bin/promo_v3). The predicted binding sites of E2F5 to miR‐106a‐5p were first confirmed using luciferase reporter assays (Figure 6a–c). Under the treatment of miR‐106a‐5p mimics, both E2F5 protein and mRNA levels were significantly reduced in PDLSCs, whereas they were increased with miR‐106a‐5p inhibitor (Figures 6d and S3A). During osteogenic induction in PDLSCs, the mRNA level of E2F5 gradually increased, and negatively correlated with the level of miR‐106a‐5p (Figure S3B,C). While lncPCAT1 seemed to positively regulate E2F5 expression in PDLSCs (Figure S3D,E). RIP‐Ago2 assay also confirmed that lncPCAT1 could also inhibit the binding of E2F5 to RISC (Figure 6e,f). lncPCAT1 functions as a molecular sponge for miR‐106a‐5p to facilitate expression of E2F5 were then confirmed (Figure S3F,G). The impacts of E2F5 on osteogenic process were subsequently evaluated. Inhibition of E2F5 led to decreased osteoblast‐related genes at protein and mRNA levels (Figures 6g and S3H). ALP activity assay as well as ARS and ALP staining confirmed the promotion of E2F5 on osteogenesis (Figure 6h,i). In vivo experiment, H&E and Masson staining further verified silence E2F5 led to increased osteoid formation (Figure 6j).

The article "A feed‐forward regulatory network lncPCAT1/miR‐106a‐5p/E2F5 regulates the osteogenic differentiation of periodontal ligament stem cells" was retracted in 2023. Reasons: errors in the images; duplicated images; unreliable results or conclusions.

**Figure 6:** E2F5 could also promote osteogenesis under the regulation of lncPCAT1/miR‐106a‐5p. (a) Schematic diagram of the miR‐106a‐5p putative binding sites in wild‐type and mutant E2F5 3′‐UTR. (b and c) The binding sites of miR‐106a‐5p to wild‐type or mutant E2F5 3′‐UTR under transfection of miR‐106a‐5p mimics or inhibitor were determined with luciferase reporter assay (*n* = 3). (d) The protein level of E2F5 in PDLSCs transfected with miR‐106a‐5p mimics or inhibitor was determined by Western blot analysis. (e, f) RIP assay of the enrichment of Ago2 on lncPCAT1, E2F5 transcripts relative to IgG in PDLSC cells transfected with lncPCAT1 overexpression or silence lentivirus and their corresponding controls (*n* = 3). (g) The protein levels of E2F5, RUNX2, OSX, and BMP2 in PDLSCs transfected with sh‐E2F5 at 7 days after osteogenic induction were determined by Western blot analysis. (h, i) Osteogenic differentiation of PDLSCs transfected with sh‐E2F5 was determined by ALP activity, ARS and ALP staining. (j) H&E and Masson staining were performed in E2F5‐silenced PDLSCs in vivo (*n* = 5 per group). Data represent mean ± *SD*. *p  < 0.05, **p  < 0.01, ***p  < 0.001. 3′‐UTR: 3′‐untranslated region; Ago2: argonaute 2; ALP: alkaline phosphatase; BMP2: bone morphogenetic protein 2; IgG: immunoglobulin‐G; lncPCAT1: prostate cancer‐associated ncRNA transcript‐1; miR: microRNA; NC: negative control; OSX: osterix; PDLSCs: periodontal ligament stem cells; RIP: RNA‐binding protein immunoprecipitation; RUNX2: Runt‐related transcription factor 2 [Color figure can be viewed at wileyonlinelibrary.com]

### 3.7 E2F5 formed a feed‐forward regulatory network together with lncPCAT1/miR‐106a‐5p

Regulatory feed‐forward loops have been reported to involve in many biological process (Chen et al., 2015; Fang et al., 2016; Szekeres et al., 2014). Whether E2F5 could function as a regulator of lncPCAT1 remained to be elucidated. Bioinformatics predicted that E2F5 might bind to the promoter of lncPCAT1 (Figure 7a). Therefore, we conducted luciferase reporter assay and confirmed this result (Figure 7b). Consistently, ChIP assay showed that E2F5 could directly bind to the predicted binding site (BD; Figure 7c,d). Under E2F5 inhibition, downregulated lncPCAT1 along with upregulated miR‐106a‐5p were observed (Figure 7e), indicating a potential feed‐forward regulatory network on osteogenic differentiation.

The article "A feed‐forward regulatory network lncPCAT1/miR‐106a‐5p/E2F5 regulates the osteogenic differentiation of periodontal ligament stem cells" was retracted in 2023. Reasons: errors in the images; duplicated images; unreliable results or conclusions.

**Figure 7:** E2F5 formed a feed‐forward regulatory network together with lncPCAT1/miR‐106a‐5p. (a) Putative binding sites of E2F5 to the promoter of lncPCAT1 were predicted using PROMO database. (b) The binding sites of E2F5 to the promoter of lncPCAT1 were determined by luciferase reporter assay (*n* = 3). (c, d) ChIP assay of the enrichment of E2F5 on lncPCAT1 promoter relative to IgG in PDLSC cells (*n* = 3). A random region without binding site acted as a negative control (NEG). (e) The levels of lncPCAT1 and miR‐106a‐5p in E2F5‐silenced PDLSCs were determined by RT‐qPCR (*n* = 3). Data represent mean ± *SD*. *p  < 0.05, **p  < 0.01, ***p  < 0.001. BD: binding site; ChIP: chromatin immunoprecipitation; IgG: immunoglobulin G; lncPCAT1: prostate cancer‐associated ncRNA transcript‐1; lncPCAT1: prostate cancer‐associated ncRNA transcript‐1; miR: microRNA; NC, NEG: negative control; PDLSCs: periodontal ligament stem cells; RT‐qPCR: reverse transcription quantitative polymerase chain reaction [Color figure can be viewed at wileyonlinelibrary.com]

## 4 DISCUSSION

Loss of osteogenic potential of PDLSCs under stimulations such as hypoxia and inflammation may partially lead to the loss of supporting periodontal tissues. It was reported that PDLSCs cultured under hypoxia exhibited decreased osteogenic potential as well as deceased expression of Oct‐4 and SOX2 through downregulation of ERK 1/2 pathway (Mohyeldin, Garzon‐Muvdi, & Quinones‐Hinojosa, 2010; Y. Zhou, Fan, & Xiao, 2014). Determination of the core regulation of osteogenesis could further facilitate our understanding of the impaired osteogenic potential of PDLSCs under hypoxia or inflammation. In our study, we confirmed lncPCAT1 was increased during osteogenic induction (Figure 1) and found that overexpression of lncPCAT1 in PDLSCs led to significantly increased osteogenesis both in vivo and in vitro, while inhibition of it led to decreased osteogenic potential of PDLSCs (Figure 2), indicating a potential role of lncPCAT1 in regulation of osteogenesis in PDLSCs.

Previous studies have shown the important role of lncPCAT1 in tumorigenesis and tumor progression. Shen et al. (2017) found that the expression level of lncPCAT1 was significantly higher in patients afflicted with multiple myeloma (MM), indicating its role as a potential biomarker in MM. It was also demonstrated that lncPCAT1 could sponge miR‐122 and therefore inhibited the Wnt/β‐catenin signaling pathway and the tumor progression in extrahepatic cholangiocarcinoma (F. Zhang et al., 2017). But there was no research considering the effect of lncPCAT1 on osteogenic differentiation, and our study revealed for the first time that lncPCAT1 could positively regulate the osteogenesis in PDLSCs. Considering the sponge effect of lncPCAT1, we further explored the underlying interaction between lncPCAT1 and miRNA.

The article "A feed‐forward regulatory network lncPCAT1/miR‐106a‐5p/E2F5 regulates the osteogenic differentiation of periodontal ligament stem cells" was retracted in 2023. Reasons: errors in the images; duplicated images; unreliable results or conclusions.

MiR‐106a is a member of the miR‐17 family. It involved in several biological properties of cancer cells such as cell viability, apoptosis and chemoresistance (Pan, Zhuang, Zheng, & Pei, 2016). With regard to its effect on osteogenic differentiation, it was shown that miR‐106a was downregulated in mesenchymal stem cells treated with BMP2 (Li et al., 2008) Manochantr and so forth found that miR‐106a was also downregulated during the osteogenic differentiation of mesenchymal stem cells derived from amnion, while anti‐miR‐106a could promote the osteogenic process (Manochantr et al., 2017). Analysis on LncRNABase and NONCODE revealed that PCTA1 could bind to miR‐106a‐5p, and the binding sites were confirmed by luciferase reporter assay (Figure 3b,c). Moreover, lncPCAT1 could sponge miR‐106a‐5p and modulate its effects on osteogenic induction (Figure 4g‐j), indicating the possible involvement of a lncRNA‐miRNA regulatory network during osteogenic differentiation.

The target genes of miR‐106a‐5p were further investigated. It has been previously reported that BMP2 is the direct target of miR‐106a, and upregulation of miR‐106a led to suppression of BMP2 level (Li et al., 2013). BMP2 is an important differentiation‐inducing factor that induces the osteogenesis and bone regeneration in PDLSCs (Bais et al., 2009; Oliveira, Martins, Lima, & Gomes, 2017). The Smad family members can further mediate the osteogenic induction effect of BMPs (Hata et al., 2000; Yoshida et al., 2000). Following activation of BMP receptor II by BMP2, both Smad1, Smad5 and Smad8 are activated and translocate to the nucleus forming a complex with Smad4, therefore activate the transcription of several genes and regulate the cell differentiation (Urata et al., 2018).

Moreover, we unraveled for the first time that E2F5 could regulate osteogenesis through targeting the promoter of lncPCAT1. Mammal E2F transcription factors family comprises of 8 genes that together promote cell cycle‐related genes and regulate cell proliferation (Attwooll, Lazzerini Denchi, & Helin, 2004; Chen, Tsai, & Leone, 2009; Zhan et al., 2014). It has been reported that E2F5 could be regulated by several miRNA, including miR‐154‐5p and miR‐98 (Cai, Huo, Wang, Chen, & Yang, 2017; Yao et al., 2013; Zheng et al., 2017). Consistent with previous report, we confirmed that miR‐106a‐5p could inhibit the expression of E2F5, while lncPCAT1 could sponge miR‐106a‐5p to protect E2F5 from that inhibition. Furthermore, E2F5 could bind to the promoter of lncPCAT1 and promote its expression, forming a feed‐forward lncPCAT1/miR‐106a‐5p/E2F5 regulatory network targeting BMP2 and osteogenesis (Figure 8). It was the first report to consider the effect of E2F5 on osteogenesis, and it provided a novel regulatory network on osteogenic differentiation.

The article "A feed‐forward regulatory network lncPCAT1/miR‐106a‐5p/E2F5 regulates the osteogenic differentiation of periodontal ligament stem cells" was retracted in 2023. Reasons: errors in the images; duplicated images; unreliable results or conclusions.

**Figure 8:** Schematic diagram of the regulation of osteogenesis through the lncPCAT1/miR‐106a‐5p/E2F5 regulatory feed‐forward loop targeting BMP2. BMP2: bone morphogenetic protein 2; lncPCAT1: prostate cancer‐associated ncRNA transcript‐1; PCAT1: prostate cancer‐associated transcript‐1; miR: microRNA [Color figure can be viewed at wileyonlinelibrary.com]

## 5 CONCLUSION

Considering minority of the ncRNAs have been functionally determined, the regulation of biological functions by lncRNA‐miRNA interaction networks may be far more important as we previously considered. In our study, we identified the regulation of osteogenic potential of PDLSCs with a feed‐forward regulatory network composed of lncPCAT1/miR‐106a‐5p/E2F5 through regulation of several osteogenic genes, including BMP2, RUNX2, and OSX. Our study exhibited the complicated regulation within ncRNA and provided a promising target to regulate the osteogenic potential of PDLSCs for treatment of periodontitis.

### 5.1 Significance

LncRNA‐miRNA regulatory network has evolved to be a crucial regulatory element in multiple biological events, but its role has not been fully understood in osteogenic differentiation of PDLSCs. We identified that lncPCAT1 was gradually increased during osteogenic differentiation of PDLSCs and further found that lncPCAT1 could positively regulate the differentiation process both in vitro and in vivo. With bioinformatic prediction and luciferase reporter assay confirmation, we identified that lncPCAT1 sponged miR‐106a‐5p and then regulated its effect on PDLSCs during osteogenic differentiation. Moreover, we found for the first time that E2F5 could bind to the promoter of lncPCAT1, and then formed a feed‐forward regulatory network targeting BMP2, a crucial gene involved in osteogenic differentiation. Notably, our study inferred a novel lncRNA‐miRNA regulatory network on osteogenic differentiation of PDLSCs. Furthermore, we proposed that this regulatory loop could emerge as a potential target to modulate PDLSCs differentiation potential.

## CONFLICT OF INTERESTS

The authors declare that there are no conflict of interests.

## AUTHOR CONTRIBUTIONS

B. J. and X. Q. contributed the central idea, analyzed the majority of the data and wrote the initial draft of the manuscript. The remaining authors contributed to refining ideas, performing additional analyses and finalizing the manuscript.

The article "A feed‐forward regulatory network lncPCAT1/miR‐106a‐5p/E2F5 regulates the osteogenic differentiation of periodontal ligament stem cells" was retracted in 2023. Reasons: errors in the images; duplicated images; unreliable results or conclusions.

## Supporting information

Supporting information
